# Tractor Cab Ergonomics Optimization Based on the Simplified Model of Upper Limb from the Perspective of Public Health

This article has been retracted.

**DOI:** 10.1155/2022/2411301

**Published:** 2022-08-02

**Authors:** Fei Yang, Nian Wang, Min Kang, Haoying Wang, Meng Wang

**Affiliations:** College of Engineering, Nanjing Agricultural University, Nanjing 210031, China

## Abstract

The study of tractor ergonomics is both an essential part of public health and a very significant part of the scientific community's focus at the moment. It offers a foundation for the layout design of the tractor cab, making it possible to effectively avoid occupational diseases, minimize the number of safety accidents, and enhance the comfort of operation. Devices are categorized as control rod devices, knob-type devices, and steering wheels according to the various modes of operation of the tractor cab. Steering wheels are also included. The ease of handling of a number of different components was ranked according to how well they performed on the fast evaluation approach for the upper limbs. After that, in accordance with the concept that underpins this evaluation approach, the comfortable range of motion of human upper limb joints is evaluated while undergoing a variety of manipulation modalities. In conjunction with the structure of the human body and the characteristics of its movement, a streamlined point-line structure model of the human upper limb is constructed, with the H-point serving as the reference point. The problem of figuring out how to distribute the control components in the best possible way has been solved, and the optimal distribution range diagram of the steering wheel has been obtained. The ideal height for the distribution of control rod devices is around 300–400 millimeters, whereas the ideal height for the distribution of knob-type devices is approximately 200–500 millimeters. In conclusion, the cab design of the KAT2204 tractor is improved upon thanks to the analysis done in this study, which can be found above. The legitimacy of the research conclusion is confirmed by the fact that the RULA value is lower than 2, which is proved by the fact that the design findings are validated by the Creo Manikin module. The ergonomics of the tractor cab were taken into consideration when using this research approach as a reference.

## 1. Introduction

The tractor is a kind of heavy machinery with a poor working environment and complex control system. Every element in its cab design and the man-machine system design related to the cab is related to the normal and efficient operation of the machinery and the safe and comfortable control of the driver. Therefore, in the industrial design of the tractor, the appeal of the humanization concept is particularly prominent [1]. In the study of the tractor cabs, Henry Dreyfuss, an American industrial designer, is regarded as the first person to study tractor ergonomics. In 1950, when Henry Dreyfuss designed the tractor cab for John deer company, he applied the ergonomic design theory in the aircraft pilot ship to the design of control rod devices in the tractor cab, distinguished the control handle by color and shape, and designed it as a standardized part produced by the assembly line [2]. With the development and improvement of ergonomics theory, the seat, display device, control device, driving environment, and safety performance of tractor cab have been deeply studied [3–6].

Tractor cab ergonomics research is one of the key fields of public health. For example, in the U.S.; one of the public health focuses is the effectiveness of rollover protective structures for preventing injuries associated with agricultural tractors because agriculture ranks fourth among U.S. industries for work-related fatalities. Relevant studies include seating discomfort and operating comfort of tractor cabs [7], and the design and development of tractors need to consider how to reduce safety accidents during operation [8] and prevent occupational diseases of tractor drivers [9]. The weakness of basic research on the man-machine of the tractor cab and the lack of cab design basis and optimization methods restricts the comfort of tractor operation. At the same time, it is necessary to reduce safety accidents during operation and prevent occupational diseases of tractor drivers.

At present, the world has focused on the research of cab and seat damping suspension [10, 11]. The research on ergonomics of tractor cabs in China started relatively late, mostly focusing on theoretical analysis [12, 13]. It can provide a valuable reference for the cab design by using the digital method to carry on the ergonomics research to the tractor cab [14]. At present, the virtual reality assessment system [15] and the field of vision, driving computer-aided system [16] have been used to study the cab ergonomics. RULA (Rapid Upper Limb Assessment [17]) is an important research method of ergonomics based on the risk assessment of muscle imbalance published by Dr. Lynn and Dr. Nigel Corlett of Institution of Occupation Efficiency in 1993, University of Nottingham. This method has been widely used in the development of various products after developments and applications, such as ergonomics evaluation of aircraft maintenance tasks [18], efficiency research of tables and chairs [19], and the research combination of free modulus magnitude estimation [20], which all provide ergonomical references for the design and development of products, as well as the development of the evaluation for finger disorders and an evaluation method based on a load of upper limb based on the core idea of RULA evaluation method [21].

The RULA evaluation method is used for the spatial arrangement of the tractor cab control device in this research. The document can be found here. In conjunction with the RULA evaluation system, an examination of the operating characteristics of each control part of the tractor cab, such as its mode of operation and frequency of use, is carried out. The range of motion of each joint was evaluated using the RULA assessment system, and a mathematical model of the human upper limb was constructed. The last step is to use MATLAB software to do a simulation of the experiment so that we can determine the ideal size of each control device. According to the size range, it may be used to influence the design of the control platform within the tractor cab, improve the comfort and accuracy of the driver, and offer a reference for the study of the ergonomics inside the cab.

## 2. Analysis of Cab Control Components

### 2.1. Factors Affecting the Status of Upper Limb Disorders

In RULA, the main influence factors of the upper limb disorders are the angle of each joint, when each joint is in the right-angle position, the human body muscle disorder is the smallest. However, apart from the influence factors of the joint, the manipulation of the device will also affect the comfort of the driver [22].

At each point within its range, the human wrist is capable of a substantial degree of torsion. When working, the wrist will be in the position that provides the greatest level of comfort when it is in the middle position of the torsional range. On the other hand, if the wrist is in a limited position, there is a greater risk of dislocation. In the actual work, depending on the actual needs of the circumstance, it may occasionally require the staff to maintain an action for a long period or it may require them to frequently repeat an action. Both of these requirements can be addressed by doing the same action. Because of this, there is an increased possibility that employees would develop muscular diseases; hence, it is essential to have distinct conversations about the various kinds of equipment. In addition, it is essential to keep in mind that the potential for developing a muscle problem is influenced in a manner that is distinct for each type of device.

Additionally, during the course of the real work, the staff may occasionally be forced to bear a certain load. The condition of the legs will also affect how comfortable the task is for the individual. Because the driver is not required to carry weight in the usual working condition of the cab, the risk that would be caused by carrying a load in the scenario, that is, the focus of this study is not taken into account. This is because the driver is not obliged to carry weight.

### 2.2. Analysis of Cab Control Devices

The ergonomic design of the tractor cab is mainly based on the operator's physiological characteristics, sports characteristics, psychological characteristics, physical limits, habits, and other factors, combined with the ergonomic design principles, to reasonably design the structure of control rod devices, display adjustment devices and seats in the tractor cab, minimize the noise and vibration in the cab [23], and provide a convenient and comfortable working environment for the driver [24, 25]. This paper takes the high-power wheeled tractor (about 200 HP tractor) as the main research object and analyzes the layout and design dimensions of the tractor cab. From the perspective of ergonomics, the components in the tractor cab can be divided into five categories: hand control components, foot control components, visual display components, driving seat, and driving space [26].

The composition of the cab of general tractors is shown in Figure 1. According to the different modes of operation, and taking the above influencing factors into account, control devices in the cab are classified into lever devices, knob devices, and steering wheels. The risk of imbalance when operating is ranked as level 0 is the minimum and level 2 is the maximum, and the operating devices are summarized are shown in Table 1.

### 2.3. Evaluation of Operating Comfort

The RULA is a method that evaluates designs on the basis of muscular disorders; the final score is used to determine whether or not a design is reasonable; if the final score is 1 or 2, the design may be accepted. Rating of the limb disorders, rating of the trunk disorder, and the final score are the three elements that make up the RULA evaluation technique. The final score section is a summary of the first two parts and rates the disorders by synthesizing the risk level of muscular disorder in certain settings. When building the model of the upper limb and solving the problem, the trunk's backward-inclined angle is less than 10° since the body does not lean forward very often when the conditions are those of a tractor cab. After conducting score screening according to the rating criteria of each portion, it will eventually be possible to attain a pleasant moving angle for each joint. Take the vertically downward direction as the 0° position when the control object is the steering wheel. The motion range of the shoulder can be obtained for the upper lift, which is 0° to 20°, and the intersection angle of the upper arm and the forearm is 60° to 100°. When the control object is of the knob type, the motion range of the shoulder can be obtained as 0° to 100° for the upper lift, and the upper arm and forearm intersection angle can be 0° to 100° as well. When the control object is a device of the joystick variety, the motion range of the shoulder can be obtained as 0° to 45° for the upper lift, and the upper arm and forearm intersection angle can range from 0° to 100°.

## 3. Establishment and Solution of the Simplified Model of the Upper Limb

### 3.1. Establishment of the Upper Limb Model

In the analysis of the operating device size range, it needs to combine with the characteristics of the structure of the human body and its movement to calculate the placement range of operating devices, in consideration of the spatial arrangement of the control device, the shoulder width, and turning angle range of the body should also be taken into consideration. Combined with the D-H model commonly used in multirigid body kinematics, wearable robots established the D-H model of human upper limb motion which is used to analyze the human upper limb motion [27]. Based on the basic idea of the D-H model, the human body model is transformed into the point-line structure whose each point represents a joint and line for the skeleton, as is shown in Figure 2. Then, take the hinge H point of the human body and the thigh as the axis origin, the tractor driving direction as *X*-axis direction and *Y*-axis direction is upward perpendicular to the ground, establishing the plane coordinate system. H point is hip point, which is in the human body template for the hip joint [28]. In the cab working conditions, when the driver operating all kinds of operates devices, the hip joint position relative to the cab is stationary, so take the H point as the origin of coordinates of the mathematical model for the analysis of human upper limb movement is convenient. And, according to the results of the design of the cab, as long as the spatial position of the H point can be determined, it can be conveniently used to transform the Cartesian coordinate system and then guide the design work. The simplified point-line structure is shown in Figure 2. The coordinates of the location of points can be calculated according to the geometric relations, of which *θ*_1_ represents the body's backward-inclined angle, *θ*_2_ represents the human upper arm lift angle, and *θ*_3_ refers to the angle between the forearm and upper arm extension lines.

### 3.2. Size Solution of the Joystick and Knob Device

The joystick and knob type devices are generally distributed in the side way of the driver, part of the control devices in operation even require the driver's small turn. So, in the optimization calculation of the handling device, it also needs to add the relevant parameters based on the original mathematical model.  Figure 3 is a top view of the human upper limb model, namely, observing the mathematical model of the line structure along the *Y*-axis direction, which *θ*_4_ refers to two of the body's shoulder line and the *Z*-axis angle, namely, the torsion angle of the human body; *θ*_5_ refers to the human arm stretching angle. *l*_1_, *l*_2_ ,  *l*_3_ ,  and *l*_4_ refer to shoulder height, upper arm length, forearm length, and unilateral shoulder width of the human body, respectively.

According to the mathematical model established above, the position of the target point is calculated, and it is known that the operating angle of each part of the body is shown in Table 2.

In the solution of three-dimensional coordinates of target points, the driver is determined to be at an angle of *θ*_1_ firstly and then raise the upper arm and forearm when operating control rod devices and knob-type devices on the side. The angle between the upper arm and the plumb line is *θ*_2_. The lifting angle of the forearm relative to the boom is *θ*_3_. At this time, the coordinate expressions of the target points are

(1) $$\begin{array}{c} x=l_{2}\cdot \;\sin\;\theta_{2}+l_{3}\cdot \;\sin\left(\theta_{2}+\theta_{3}\right)-l_{1}\cdot \;\sin\;\theta_{1},\\ y=l_{1}\cdot \;\cos\;\theta_{1}-l_{2}\cdot \;\cos\;\theta_{2}-l_{3}\cdot \;\cos\left(\theta_{2}+\theta_{3}\right),\\ z=l_{4}. \end{array}$$

Then, the shoulder rotation and arm abduction are completed. The included angle between the connecting line of the two shoulder joints and the *Z* axis is *θ*_4_. The external rotation angle between the boom and the relative shoulder is *θ*_5_. At this time, the calculation formula of target point coordinates is derived as follows:

(2) $$\begin{array}{c} x=\left(l_{2}\cdot \;\sin\;\theta_{2}+l_{3}\cdot \;\sin\left(\theta_{2}+\theta_{3}\right)-l_{1}\cdot \;\sin\;\theta_{1}\right)\cdot \;\cos\left(\theta_{4}+\theta_{5}\right)-l_{4}\cdot \;\sin\;\theta_{4},\\ y=l_{1}\cdot \;\cos\;\theta_{1}-l_{2}\cdot \;\cos\;\theta_{2}-l_{3}\cdot \;\cos\left(\theta_{2}+\theta_{3}\right),\\ z=\left(l_{2}\sin\;\theta_{2}+l_{3}\sin\left(\theta_{2}+\theta_{3}\right)\right)\cdot \;\sin\left(\theta_{4}+\theta_{5}\right)+l_{4}\cdot \;\cos\;\theta_{4}. \end{array}$$

Five values have been taken at the same distance within *θ*_1_, *θ*_2_, *θ*_3_, *θ*_4_, and *θ*_5_, and then the values are taken into MATLAB to repeat the calculation, with the number of repeat tests 54 times. Then, the results of each calculation are mapped in the coordinates of the point, as the joystick device size optimization results are shown in Figure 4, and knob type devices size optimization results are shown in Figure 5.

The aforementioned data need to be processed in two dimensions so that the results of Figures 4 and 5 can be presented in a manner that is easier to understand. It is possible to make an educated guess about the value range of the vertical axis in the two figures by looking at Figures 4 and 5. The size optimal range scatter of control rod devices along the vertical axis is shown in Figure 4 (0, 1000). Figure 5 illustrates that the best size range for scattering of knob-type devices along the vertical axis is (0, 600). Take the average of nine segments in the range of Figure 4 from 100 to 1000, and take the average of six segments in the range of Figure 5'(s) from 0 to 600. After projecting the points from each section onto the XOZ plane, one may obtain the scatter diagram for the height section that corresponds to that section. The best range of control rod devices for the side console at the equivalent height is the range that corresponds to the scatter dispersion range. Both Figures 6 and 7 display the scatter plots that were generated as a result.

Within this height range, the ideal distribution space for the horizontal space can be seen to be reflected by the position of the points on the outermost and surrounding areas of the scatter diagram. It is possible to conclude that the optimal distribution height of control rod devices is approximately 300–400 millimeters, followed by 200–300 millimeters and 400–500 millimeters, and that the optimal distribution height of knob devices is 200–500 millimeters by observing the area that is surrounded by the points that are further out.

### 3.3. Solution of Steering Wheel Size

According to the criteria of the forearm imbalance rating, the forearm imbalance rating level will increase when the current working position of the arm is over the human body's symmetry surface or when the arm is working outside the body. This is because these positions cause the forearm to be out of alignment with the rest of the body. This criterion can demonstrate that the design of the steering wheel location should ideally be in the plane of body symmetry and that the wheel diameter should be about equivalent to the width of a human shoulder. As a result, there is a two-dimensional zone on the human body that constitutes the ideal placement for the steering wheel. Given the situation that the steering wheel is a special control device, the mathematical model can be simplified to improve the efficiency of the analysis and make the optimization results more intuitive.

In order to facilitate the solution of the position of the target, the human body model is simplified into a point-line structure, where each point represents the joint and line represents the skeleton, and then take H point as the origin of coordinates, the tractor driving direction as *X*-axis direction, and *Y*-axis direction is upward perpendicular to the ground, establishing the plane coordinate system. The simplified point-line structure is shown in Figure 8, and the coordinates of the target points can be obtained according to the geometric relations:

The simulation test is conducted by using MATLAB software programming, and the optimal range is covered as far as possible. The range of motion angle of each joint is as follows while the driver is operating the steering wheel, where *φ*_4_ is set for the convenience of calculation:

(3) $$\begin{array}{c} \varphi_{1}\in 0^{o}，10^{o},\\ \varphi_{2}\in 0^{o}，20^{o},\\ \varphi_{3}\in 60^{o}，100^{o},\\ \varphi_{4}=180^{o}-\varphi_{2}-\varphi_{3}. \end{array}$$

According to the geometric relations, the calculation formula of the coordinates of the target points can be deduced as follows of which *l*_1_, *l*_2_,  and *l*_3_ are shoulder height, upper arm length, and forearm length, respectively:

(4) $$\begin{array}{c} x=-l_{1}\cdot \;\sin\;\varphi_{1}+l_{2}\cdot \;\sin\left(\varphi_{1}+\varphi_{2}\right)+l_{3}\cdot \;\sin\;\varphi_{4},\\ y=l_{1}\cdot \;\cos\;\varphi -l_{2}\cdot \;\cos\left(\varphi_{1}+\varphi_{2}\right)+l_{3}\cdot \;\cos\;\varphi_{4}. \end{array}$$

We took 10 values at the equal distance within the scope of *ϕ*_1_, *ϕ*_2_, and *ϕ*_3_ and then calculated repeatedly in MATLAB; the number of repeat tests was 10^3^ times. Then, the results of each calculation are plotted in the coordinate system, and the results are shown in Figure 9.

## 4. Design and Verification Based on Pro/E Manikin

### 4.1. Layout Optimization of the Control Device

According to the optimization results obtained by the method described above, an optimization design of a cab layout based on a KAT2204 type tractor was taken as the design object for optimization. The primary areas of the cab that were targeted for optimization were the reversing lever, hand throttle, gear handle, multifunction joystick, and steering wheel.  Figure 10 demonstrates the establishment of a rectangular coordinate system with the H point serving as the origin.  Table 3 provides information regarding the relative position and size of the various important components.

### 4.2. Display of Simulation Results

A plug-in component known as Manikin is included in the engineering modeling program known as Pro/E. This component can be utilized to carry out the associated ergonomics analysis by invoking a human body model. It has the ability to assess people's levels of comfort when they perform certain actions based on RULA. Built the model of the optimized layout of the cab and analyzed the RULA values of operating relative devices by calling the human body model; the analysis results are shown in Figure 11; each RULA value of the operating member is not greater than 2, so the analysis method is feasible and effective, and the results obtained can provide a valuable reference for the design of the cab. Figure 11 shows the results of the analysis.

## 5. Conclusion

The conclusion of our work can be summarized as follows:

1. This work provides an analysis of the primary components and research methodologies used in the ergonomics design of the tractor cab. It also proposes a strategy for optimizing the ergonomics of the tractor cab layout based on a simplified model of the upper limb from the point of view of public health.
2. The angle of joint movement under specified situations was selected by the RULA evaluation method, and the simplified model of the human upper limb was constructed based on the D-H model of the human upper limb that was proposed by wearable robots. MATLAB was used to carry out several rapid simulation experiments in order to obtain the optimal range of the operating parts, as well as the optimal design height of the side console. H point was used as the origin of the rectangular coordinate system. H point was used as the origin of the rectangular coordinate system.
3. According to the optimization results obtained by the Manikin module, the results are less than or equal to 2, which can be verified that the optimization results presented in this paper were feasible and effective.

The RULA assessment method is capable of being utilized for the purpose of conducting an ergonomic study under certain circumstances. The results of an ergonomic study conducted on a tractor cab using the Pro/E Manikin module have demonstrated that the findings are capable of being disseminated and utilized. This method not only serves as a reference for the investigation of the ergonomics of tractor cabs but also establishes the groundwork for the further improvement of tractor cabs.

## Figures and Tables

**Figure 1:** Component division in the tractor cab.

**Figure 2:** Point-line model of the human upper limb.

**Figure 3:** Top view of the point-line model of the human body.

**Figure 4:** Size optimal range scatters diagram of control rod devices.

**Figure 5:** Size optimal range scatter diagram of knob-type devices.

**Figure 6:** The optimal distribution of control rod devices at the height of 100–900 mm.

**Figure 7:** The optimal distribution of knob type devices at the height of 0–600 mm.

**Figure 8:** Simplified mathematical model of the human upper limb.

**Figure 9:** The optimum range of the steering wheel size.

**Figure 10:** Schematic diagram of the cab optimization design coordinate system. (a) Cab top view. (b) Cab side view.

**Figure 11:** Validation results of the manikin. (a) Manipulate the steering wheel. (b) Manipulate the gear lever. (c) Operate the side console. (d) Operate the front console.

**Table 1:** Induction of control device of the tractor cab.

Control device	Muscle disorders rating	Wrist disorders rating
Steering wheel	1	1
Control lever class	0	1
Knob class	0	2

**Table 2:** Joint angle parameter table (part).

Angle parameter	Control level device	Knob device
*θ*1	0^*o*^，10^*o*^	0^*o*^，10^*o*^
*θ*2	0^*o*^，100^*o*^	0^*o*^，45^*o*^
*θ*3	0^*o*^，100^*o*^	0^*o*^，100^*o*^
*θ*4	0^*o*^，20^*o*^	0^*o*^，100^*o*^
*θ*5	0^*o*^，90^*o*^	0^*o*^，100^*o*^

**Table 3:** Relative position dimensions of control devices.

Code	Control device	Position coordinate
A	Steering wheel	(0, 354, 320)
B	Hand throttle	(210, 450, 25)
C	Main gear shift lever	(315, 334, 90)
D	Auxiliary gear lever	(360, 300, 90)
E	Power output switch	(327, 39, −177.6)
F	Refrigeration knob	(310, −280, 180)
G	Heating knob	(300, −340, 180)

## Data Availability

The dataset used to support the findings of this study are available from the corresponding author upon request.
